# Finite Element Analysis and Comparative Study of 4 Kinds of Internal Fixation Systems for Anterior Cervical Discectomy and Fusion in Children

**DOI:** 10.1155/2022/6072927

**Published:** 2022-07-11

**Authors:** Ziyu Li, Jianqiang Zhou, Xingyue Qu, Shaojie Zhang, Xiaoyan Ren, Xing Wang, Kun Li, Zhijun Li, Shang Gao, Xiaohe Li

**Affiliations:** ^1^Graduate School of Inner Mongolia Medical University, Hohhot, Inner Mongolia 010110, China; ^2^Department of Orthopedics, Hohhot First Hospital, Hohhot, Inner Mongolia 010000, China; ^3^Department of Human Anatomy, School of Basic Medical Sciences, Inner Mongolia Medical University, Hohhot, Inner Mongolia 010110, China; ^4^Department of Endocrinology, Affiliated Hospital of Inner Mongolia Medical University, Hohhot 010050, China; ^5^Digital Medical Center, Inner Mongolia Medical University, Hohhot, Inner Mongolia 010110, China

## Abstract

**Background:**

Spinal injury in children usually occurs in the cervical spine region. Anterior fixation of the lower cervical spine has been applied in treating pediatric cervical spine injury and disease due to its stable and firm mechanical properties. This study performed finite element analysis and comparison of four different anterior cervical internal fixation systems for children to explore more standard methods of anterior cervical internal fixation in children and seek more effective and safe treatment for children's cervical spine diseases.

**Methods:**

A finite element model of 6-year-old children with lower cervical spine C4/5 discectomy was established, and the self-designed lower cervical spine anterior locking internal fixation system ACBLP and the children's anterior cervical internal fixation system ACOP, ACVLP, and ACSLP plate screws were fixed and loaded on the model. 27.42 N·m torque load was applied to each internal fixation model under six working conditions of anteflexion, backward flexion, left flexion, right flexion, left rotation, and right rotation, to simulate the movement of the cervical spine. The activity and stress distribution cloud diagram of each finite element model was obtained to explore the optimal method of anterior cervical fixation in children.

**Results:**

In the four internal fixation models of ACOP, ACVLP, ACSLP, and ACBLP, the mobility of the C4/5 segment showed a decreasing relationship, and the mobility of adjacent segments increased significantly. In the Mises stress cloud diagram of the cervical spine of the four models, the vertebral body and accessories of the ACBLP model born the least stress, followed by ACSLP. The steel plate and screws in the ACVLP internal fixation model were the most stressed. The stress of the internal fixation system (plate/screw) in all models increased in the order of ACBLP, ACSLP, ACVLP, and ACOP.

**Conclusions:**

ACBLP internal fixation system had obvious advantages in anterior internal fixation of the lower cervical spine in children, C4/5 had the smallest degree of movement, relative displacement was minimal, and the stress on the centrum and pedicle was the least, while the stress on the plate screw was relatively the smallest.

## 1. Introduction

Cervical spondylosis is a progressive degenerative disease of the intervertebral disc and adjacent vertebrae, which can cause neck pain, radiculopathy, and myelopathy. Maintaining stability after cervical spine surgery is a challenging problem [1]. The continuous improvement of anterior, posterior, and combined approaches to cervical spine internal fixation plays an increasingly important role in treating cervical spine injuries and diseases [2]. Cloward [3] first used the cervical plate and screw internal fixation system for anterior cervical interbody fixation in 1964 to improve the mechanical stability of cervical lesions after surgery. Anterior plate construct is considered one of these for maintaining cervical spine stability, promoting intervertebral fusion, and reducing intervertebral dislocation after anterior cervical discectomy and fusion in subsequent clinical treatment. Some scholars conducted experimental research on the relevant mechanics of the anterior cervical plate screw internal fixation system [4–6]. Zhao et al. [7] believed that the locking independent fusion cage was more effective than the anterior plate internal fixator in the anterior cervical discectomy and fusion. Feng et al. [8] compared the mechanical properties of the cross nails and parallel nails in the anterior cervical plate screw system. It was found that there was no significant difference in the maximum pull-out force and fatigue strength of the two steel plates. However, the cross nails were more conducive to the operation, with the internal fixation effect not weakening. These studies all suggest that cross nails and locking fusion are more suitable for anterior cervical treatment. In addition, most current studies are based on adult cervical spine models, but children's cervical spine is flatter and thinner than adults, and the vertebral arch is narrower and thinner, and it is challenging to screw simultaneously difficult to insert 2 pedicle screws at the same time, and the patient's postoperative recovery is poor. Traditional anterior cervical internal fixation systems (ACOP, ACVLP, and ACSLP) have played a significant role in diagnosing and treating adult cervical spine diseases. Still, the application of such methods in children with fragile bones remains to be discussed. To solve the problem of the stability of the child's nail placement, combined with the currently used anterior cervical ORION internal fixation system, this study designed an anterior cervical bicortical pedicle locking plate (ACBLP) and established an unstable three-dimensional finite element model for children's cervical C4/5 discectomy, performed finite element analysis on this internal fixation method and other three different internal fixation methods, compared the mobility and vertebral body and accessories stress-strain of the four internal fixation methods, and explored better clinical internal fixation treatment for neck injuries in children.

## 2. Methods

### 2.1. Experimental Data

In 2019, in the Digital Medicine Center of Inner Mongolia Medical University, the finite element analysis of 4 different internal fixation methods for the child's anterior cervical approach was completed. The experimental specimen came from the corpse of a 6-year-old girl from the Anatomy Laboratory of Inner Mongolia Medical University, with a height of 115 cm and weight 41 kg. An X-ray of the cervical spine was taken to exclude cervical vertebra deformity, trauma, tumor, etc. The CT (United States, GE, Lightspeed dual-source 64-slice spiral CT) scan range was a spiral axial scan of the whole cervical spine from top to bottom. Scanning parameters are as follows: tube voltage 120 kV, tube current 125 mA, layer thickness 0.625 mm, and no interval scanning. Complete cervical spine CT image data were obtained and saved in DICOM format. The experiment was approved by the Ethics Committee of Inner Mongolia Medical University.

### 2.2. Experimental Method

#### 2.2.1. Establish a Finite Element Model for the Removal of the C4/5 Disc of the Lower Cervical Spine in Children

CT data was constructed into a normal child C3-C7 three-dimensional finite element model by Mimics 21.0, Pro/E 5.0, Geomagic studio 2015, HyperMesh 14.0, Abaqus 6.14. Multiple unit types were used to build the model, and 361012 units and 509161 nodes were contained. The C4/5 disc removal of the model was modified into an unstable finite element model. The boundary conditions and loading conditions were the same as the full model loading conditions. In the experiment, the ligament was hidden for view convenience, but the finite element analysis results were not affected.

#### 2.2.2. Establish 4 Kinds of Internal Fixed Finite Element Models

According to the child's cervical instability model, a three-dimensional model of the internal fixation steel plate and fixed locking screw was constructed. Four kinds of internal fixation plate screws were used to construct a geometric solid model to build four personalized anterior cervical internal fixation models:

1. Anterior cervical orion plate internal fixation (ACOP) for children's anterior cervical locking internal fixation system consisted of 4 ordinary vertebral screws with connected and fixed steel plates. The screws were directly driven into the vertebral body
2. Anterior cervical vertebral locking plate (ACVLP) included 4 vertebral screws with threaded heads and corresponding locking plates which is inserted into the vertebral body in the same way as ACOP
3. Anterior cervical single cortical pedicle locking plate (ACSLP) included 2 vertebral screws and 2 pedicle screws. Vertebral screws and pedicle screws were cross-locked of in the vertebral body
4. This study designed an anterior cervical bicortical pedicle locking plate (ACBLP) combined with the commonly used anterior cervical ORION internal fixation system. It is composed of vertebral screws and 2 full-thread bicortical pedicle screws penetrating the side block through the pedicle. The vertebral screws and full-thread bicortical pedicle screw were cross-locked in the vertebral body. At the same time, the two screw caps were double fused and locked on the steel plate

The elastic modulus, Poisson ratio, element type, and characteristic value of the implant material were inputted into the model [9] (implant titanium alloy *E* = 110000 MPa, *μ* = 0.3, tetrahedral element). The three-dimensional finite element models of the four internal fixation systems after cervical C4/5 discectomy were established, as shown in Figure 1.

#### 2.2.3. Loading Calculation of 3D Finite Element Model

The cervical vertebra screw and the vertebral screw were defined as close contact without sliding and compression deformation. Constraint boundary is as follows: The degrees of freedom of all nodes on the lower edge of the C7 cone were restricted in all directions, C3 was not subject to any restrictions, and the center of the upper edge of the vertebral body received a load that simulated the weight of the head. Assumptions are as follows: The material properties of the biological materials involved in this experiment were assumed to be continuous, homogeneous, and isotropic; there was no mutual sliding between the sections of the model under force; there was enough stability between the units; and the stress and deformation of each part of the material during the loading process were excluded. Loading conditions are as follows: A 27.42 N simulated head weight preload is applied to C3, and the additional pure moment of movement is 1.8 Nm [10]. ABAQUS finite element software was used for finite element analysis. According to the experimental methods of cervical spine movement characteristics and specimens, simulated cervical spine movement was divided into six types of movement: anteflexion, backward flexion left flexion, right flexion, left rotation, and right rotation.

#### 2.2.4. Setting and Operation of Different Working Conditions

The stress value of the model was set. A 27.42 N·m torque load was applied to simulate cervical spine movement to ACOP, ACVLP, ACSLP, and ACBLP after the cervical C4/5 discectomy internal fixation model, respectively, under 6 working conditions. Five points were randomly selected from C4, C5's superior articular process, contralateral superior articular process, bilateral pedicle, and vertebral body; the corresponding values were obtained to compare and analyze the biomechanical activity and stress changes of the four internal fixation models. At the same time, the stress distribution and strain of the steel plate and screw unit of the four kinds of internal fixation systems of the lower cervical spine in children.

#### 2.2.5. Statistical Analysis

The data were inputted into SPSS 22.0 for analysis. The data is expressed with $\bar{x}\pm s$. The same measurement parameter was compared in different internal fixation models by one-way analysis of variance (one-way ANOVA) with multisample means comparison, and *P* < 0.05 was considered a significant difference.

## 3. Results

### 3.1. Comparison of Activities of 4 Internal Fixation Models under 6 Working Conditions

After C4/5 segment fixation, the immediate stability of the segments of all internal fixation models was improved. In the research, smaller activity indicated higher stability. The internal fixation method had a noticeable effect on reducing mobility. The ACBLP internal fixation model had the advantages of good immediate stability and relatively small impact on adjacent segments than the original three internal fixation models. For the overall lower cervical spine range of motion of the four internal fixation models, ACOP>ACVLP>ACSLP>ACBLP, ACOP had significant differences with ACVLP, ACSLP, and ACBLP (*P* < 0.0001); ACBLP is the smallest, and the difference was significant compared with ACOP and ACVLP (*P* < 0.0001), see Table 1.

### 3.2. Cervical Spine Mises Stress Comparison of the 4 Internal Fixation Models under the 6 Working Conditions

As shown in the figure, different stress values corresponded to different colors (or) gray levels; at the same time, the calibration reference value was attached to the left side of the model. The range of the stress value could be judged by comparing the fit between this value and the color. There were apparent differences in the cervical spine Mises stress distribution characteristics in the ACOP, ACVLP, ACSLP, and ACBLP internal fixation models; the ACBLP internal fixation model has smaller and more dispersed stress distribution for the cervical spine, which conforms to biomechanical fixation, as shown in Figure 2.

For the overall lower cervical spine stress values of the four internal fixation models, ACOP>ACVLP>ACSLP>ACBLP, ACOP was significantly different from ACVLP, ACSLP, and ACBLP (*P* < 0.0001); ACBLP was the smallest, compared with ACVLP and ACSLP, and the difference was significant (*P* < 0.0001), see Table 2.

### 3.3. Steel Plate Screw Stress Comparison of 4 Internal Fixation Models under 6 Working Conditions

After removal of the C4/5 disc, the Mises stress cloud diagram of the steel plate screw under the six loading conditions of anteflexion, backward flexion, left flexion, right flexion, left rotation, and right rotation of different internal fixation models were shown in Figure 3. The stress of the steel plate screws of the internal fixation system in the model increased in the order of ACBLP, ACSLP, ACVLP, and ACOP. It showed that the stress of the ACOP internal fixation system was relatively concentrated, the stress of ACBLP was dispersed, and the stress concentration was not apparent, in line with biomechanical fixation.

## 4. Discussion

The study established a 6-year-old child's unstable working condition model after C4/5 disc removal. The model was used to compare and analyze stability and stress characteristics of 3 kinds of children's anterior cervical locking internal fixation systems ACOP, ACVLP, and ACSLP with the self-designed internal fixation system ACBLP. According to the analysis of the applied mechanical results, the conclusion was that under various working conditions, the ACBLP had the smallest mobility and was the most stable, while the ACOP had the worst stability. The increase in mobility of adjacent segments in the ACBLP internal fixation model was relatively small, while the increase in the mobility of adjacent segments in the ACOP internal fixation model was relatively large. The change in mobility was because of the conjunction of the vertebral screw and pedicle screw when fixing the unstable model. At the same time, the pedicle screw penetrated the double cortex and enhanced control and stability, and the cross-locking further enhanced the firmness. The self-designed internal fixation system ACBLP not only effectively targeted children's bone structure characteristics but also reasonably used the stability characteristics of vertebral body screw and pedicle screw. The combination of the two met the requirements for the safe diagnosis and treatment of the anterior cervical internal fixation system from the perspective of human anatomy and biomechanics.

The 4 internal fixation models fixed the C4/5 segment in comparing mobility under 6 working conditions. After the experiment, the immediate stability of the segment improved to varying degrees, indicating that the activity decreased in varying degrees. The results showed that the overall range of motion of the lower cervical spine was ACOP>ACVLP>ACSLP>ACBLP, and the influence of the ACBLP model on adjacent segments was relatively small. In this study, it was concluded that in the ACBLP internal fixation model, the effect of using the vertebral body screw and pedicle screw for internal fixation was better. ACBLP will ever model used in three kinds of internal fixation of a vertebral body with pedicle screw and use the whole thread double cortex pedicle screw for stability and penetrability of reinforcement, the vertebral bodies with entire thread double-crosses cortex pedicle screw locking, and steel plate with dual screw thread head of nail fixed lock. It effectively controls the range of motion of the cervical vertebra, improves the stability of the cervical vertebra, and provides feasible solutions for treating diseases that need to maintain the anatomical structure and stability of the cervical vertebra.

In the Mises stress cloud diagram of the cervical spine under 6 loading working conditions, under anteflexion and backward flexion conditions, although the stress of the cervical spine in the 4 internal fixation models was primarily concentrated in the C6 and C7 vertebral bodies and pedicles, it is evident that the pressure on the cervical spine in the ACBLP internal fixation model was relatively small and ACVLP was rather large. The study believed that because the stress concentration point was lower during anteflexion and backward flexion, the impact on the internal fixation model was relatively small, consistent with the previous research results of Wang et al. [11]. In the left and right flexion conditions, the stress of the cervical spine in the 4 internal fixation models was mostly concentrated around the C4 and C5 vertebral screw holes. For the left flexion, the ACBLP had minor stress in C4 and C5. For the right flexion, the stress on the C4 and C5 vertebral bodies of ACVLP were larger than other models. In the left and right flexion conditions, the force of the vertebral screw was more potent than the pedicle screw, which would lead to the loosening of vertebral screws after surgery. In the left and right rotation conditions, the stress of the cervical spine was distributed to each vertebral body in all the 4 models; the vertebral bodies of the lower cervical spine were relatively uniformly stressed. The influence on each vertebral body was not significant, compared with the previous 4 working conditions. The ACOP model had higher vertebral body stress, and the ACBLP model had less vertebral body stress. Under 6 loading conditions, the ACBLP internal fixation model was better than the original three internal fixation models in terms of stress on the vertebral body, pedicle, vertebral screw and pedicle screw, and the cervical vertebra was more dispersed, which was easier to protect children's cervical vertebra bone and stability.

In the Mises stress cloud diagram at the steel plate and screw, under anteflexion and backward flexion conditions, the C4 left screw of ACVLP, ACSLP, and ACBLP suffered more significant stress. The stress was concentrated at the junction of the screw head and the nail shaft. In the ACOP model, the screw stress was concentrated on the C5 vertebral screw during backward flexion. The stress change provided a possible reference for the loosening or breaking point of the screw [2, 12]. ACBLP, ACSLP, ACVLP, and ACOP steel plates were subject to increasing stress in the left and right flexion conditions. The steel plate in the ACBLP was the least stressed. In the ACOP, the stress was relatively concentrated in the middle of the steel plate. As in other models, the stress was relatively concentrated at the left side of the steel plate. In the four models, the C5 vertebral screw was relatively large. ACBLP screw stress was concentrated on the front third of the nail shaft. The reason might be that there was a slight movement between the screw and the steel plate in the ACOP model. In the left and right rotation conditions, the stress on the steel plate and screws in the four internal fixation models was relatively uniform. For the left rotation, the stress of the upper right corner and lower left corner of the steel plate was slightly higher. The stress of the internal fixation screw was basically concentrated on the upper right corner and the lower left corner screw. The stress on the steel plate in all models was more significant than the stress on the screw, showing the stress concentration of the steel plate. However, the maximum stress value of all internal fixation was 35.591 MPa (the C5 right screw right flexion condition), still much smaller than the yield strength of titanium alloy 894-3790 MPa. Therefore, it was not easy to cause fatigue fracture of the screw, and clinical fatigue fracture was relatively rare correlated with it [13–16]. Under 6 loading conditions, the ACBLP internal fixation model has the most minor and most dispersed stress distribution on the plate and screw, which is not easy to cause damage to the plate and screw and has more excellent protection for the cervical spine.

In summary, unlike adult anterior cervical discectomy and fusion with plate screw internal fixation, the children's cervical spine is not yet mature, the vertebral body is relatively flat, the pedicle is small, and it is very difficult to place pedicle screws in both pedicles in the vertebral body. The advantages of the ACBLP internal fixation system independently designed by this study are as follows: (1)Placing 1 vertebral screw and 1 double cortical pedicle screw in each vertebral body to improve the stability by cross nails and reduce the damage and destruction of the children's cervical vertebral body; (2) adding threads matching the steel plate to all screw caps, fusion locking the thread and steel plate, preventing the occurrence of withdrawal or loosening of screws after surgery; (3) for the pedicle screw, a full-threaded bicortical pedicle screw with the pedicle penetrating the lateral mass was used, compared to a single cortical pedicle screw, further increasing the holding force of the screw in the vertebral body, reducing screw slippage caused by too weak cervical spine in children; and (4) the ACBLP internal fixation model had the advantages of good immediate stability and relatively small impact on adjacent segments. ACBLP was the smallest for the overall lower cervical spine stress values and the stress of ACBLP was dispersed, and the stress concentration was not apparent. Therefore, the stability and force distribution of ACBLP and ACSLP internal fixation systems are relatively good. The ACBLP internal fixation system provides good support for the three columns of the lower cervical spine in children. The corresponding displacement of the stress on the three columns is smaller than other internal fixation models, embodying the good mechanical properties of locking pedicle screws. The ACBLP internal fixation model enjoys the advantages of good immediate stability and relatively small impact on adjacent segments. In addition, because the stress distribution of cervical vertebra and vertebral pedicle is smaller and more dispersed and the stress of plate and screw is less, it is safer to be applied in the treatment of children's cervical vertebra injury diseases. The result provides detailed quantitative reference information for preoperative planning and predicting postoperative mid- and long-term efficacy. The results of the study can be used for clinical reference.

## Figures and Tables

**Figure 1:** Three-dimensional finite element model of four internal fixation methods after removal of the C4/5 cervical disc in children. (a) ACOP. (b) ACVLP. (c) ACSLP. (d) ACBLP.

**Figure 2:** Cervical spine Mises stress cloud diagram of the four internal fixation models.

**Figure 3:** Mises stress cloud diagrams of steel plates and screws of four internal fixation systems.

**Table 1:** The motion range of the four internal fixation systems in different motion states ($\bar{x}\pm s$, mm).

Motion	ACOP	ACVLP	ACSLP	ACBLP
Ante flexion	1.98 ± 1.20	1.42 ± 0.88^a^	1.01 ± 0.61^ab^	0.74 ± 0.43^ab^
Backward flexion	5.53 ± 3.34	3.86 ± 2.39^a^	2.70 ± 1.61^ab^	1.98 ± 1.17^ab^
Left flexion	7.58 ± 4.38	5.45 ± 3.16^a^	3.19 ± 2.24^ab^	2.85 ± 1.59^ab^
Right flexion	7.90 ± 4.68	5.46 ± 3.20^a^	3.80 ± 2.09^ab^	2.83 ± 1.57^ab^
Left rotation	5.85 ± 3.68	4.26 ± 2.75^a^	3.03 ± 1.89^ab^	2.22 ± 1.33^ab^
Right rotation	5.78 ± 3.50	4.28 ± 2.51^a^	3.03 ± 1.74^ab^	2.21 ± 1.27^ab^

Note: compared with the ACOP group, ^a^*P* < 0.05; compared with the ACVLP group, ^b^*P* < 0.05; and compared with the ACSLP group, ^c^*P* < 0.05.

**Table 2:** The stress-strain range of 4 internal fixation systems in different motion states ($\bar{x}\pm s$, MPa).

Motion	ACOP	ACVLP	ACSLP	ACBLP
Ante flexion	2.48 ± 2.23	1.83 ± 1.69^a^	1.29 ± 1.16^a^	0.96 ± 0.84^ab^
Backward flexion	3.69 ± 1.39	2.66 ± 1.12^a^	1.91 ± 0.71^ab^	1.42 ± 0.53^abc^
Left flexion	4.28 ± 2.78	3.15 ± 2.08^a^	2.26 ± 1.47^ab^	1.66 ± 1.06^ab^
Right flexion	4.17 ± 2.59	3.09 ± 2.04^a^	2.24 ± 1.45^ab^	1.70 ± 1.11^ab^
Left rotation	4.28 ± 1.64	3.07 ± 1.21^a^	2.21 ± 0.89^ab^	1.61 ± 0.63^abc^
Right rotation	4.24 ± 1.77	2.95 ± 1.12^a^	2.09 ± 0.81^ab^	1.59 ± 0.64^abc^

Note: compared with the ACOP group, ^a^*P* < 0.05; compared with the ACVLP group, ^b^*P* < 0.05; and compared with the ACSLP group, ^c^*P* < 0.05.

## Data Availability

The corresponding author Shaojie Zhang can be contacted to request for the raw data.

## Abbreviations

ACOP: Anterior cervical orion plate
ACVLP: Anterior cervical vertebral locking plate
ACSLP: Anterior cervical single cortical pedicle locking plate
ACBLP: Anterior cervical bicortical pedicle locking plate.
